# Progress and Prospects of Research on Public Services in Sports in China: Analysis in the Context of Bibliometric Ecological Civilization and Social Networks

**DOI:** 10.1155/2022/9309074

**Published:** 2022-07-07

**Authors:** Xiang Zhong, Chao Jiang, Li Li, Haikui Zhou

**Affiliations:** ^1^School of Physical Education, Chaohu University, Hefei 238024, China; ^2^School of Economics and Law, Chaohu University, Hefei 238024, China; ^3^Graduate School University of Perpetual Help System DALTA, Manila 1740, Philippines

## Abstract

In order to better understand the current situation of Chinese public sports, this paper studies Chinese public sports. According to SATI3.2 statistics, 71 newsletters have published a total of 903 articles, of which 40 newsletters have one article, 19.7% of the newsletters have 2–9 books, and 17 magazines have more than 10 issues. The results show that by measuring data, we can better understand the current state of China's public services. This paper uses the method of bibliometric analysis to sort out and summarize the policies, characteristics, hotspots, and trends of China's public service field under the social network environment. The survey shows that the education sector has paid less for public entertainment in recent years. The research direction is system, equity, government procurement, interest, capital allocation, strategy, and supply chain. This paper highlights that the shortcomings of public sports research in our country: “public sports services” and “public sports services” are not integrated; there are many macrostudies on public service sports but few microstudies; there is no track and field research for special public groups. This paper puts forward research guidance for China's public sports services and, at the same time, strengthens the research on public services of different products of rural sports development, strengthens the research on the intelligence of sports public services, and strengthens the research on the role of public sports. Governments at all levels support and strengthen research on public sports service standards, strengthen research on public sports performance measurement measures, and strengthen public sports balance research.

## 1. Introduction

Since the 18th National Congress of the Communist Party of China, the state's right to serve public services has been proclaimed one after another. Public sports have become an important part of the “Thirteenth Five-Year Plan,” and public sports are increasingly popular [1]. The report of the 19th National Congress of the Communist Party of China pointed out that it is necessary to improve the level of public services, make people's lives easier, meet the needs of modern development, and seek a better life. In other words, building a perfect sports public service is not only one of the necessary conditions for people to live a better life, but also the inevitable condition for building a well-off society in an all-round way. At the same time, the report of the 19th National Congress of the Communist Party of China clearly put forward the development of sportsmanship. The power of athletics is related to public sports. Some scholars believe that improving the level of public sports is the only way to enhance sports strength [2]. Therefore, it is necessary to study public sports in China, which has played an important role in promoting sports. Based on this, from the perspective of bibliometrics, this research adopts the method of relational analysis to identify the status quo, characteristics, and hotspots of scientific research, so as to provide access for the public to play and for future public sports [3].

Taking the CNKI database as the literature retrieval platform, the retrieval subject is “sports public service” or including “public sports service”, the time is not limited, the source categories are “core journals” and “CSSCI”, and 1104 titles are retrieved. Then we browse and read the title information, delete the meeting notice, speech content, and draft notice, and finally determine 903 valid sample documents. We use software such as SATI3.2, COOC1.7, data element, and Ucinet6 to sort out the data, draw the network structure diagram through the Netdraw function of ucinet6, reflect the research hotspots in this field, and master the main characteristics and laws of the research as a whole [4].

The sports industry is an industry involving the national economy and people's way of life. Encouraging everyone to participate in sports and improving the national physical quality has always been the focus of the government's work. In the new business environment, the sports industry and the sports industry have become important growth drivers. The development of China's sports industry has gone through several stages of development, as shown in Figure 1.

## 2. Literature Review

Xiao L. and others said that great achievements had been made in the research of sports public service, but there are still some deficiencies [5]. Wu D., through literature review, found that the concept expression of sports public service and public sports service is not unified [6]. Even in the same article, the two concepts are mixed. However, from the perspective of Chinese expression habits, sports is used as a modifier to modify public services, which means that public services are limited to the field of sports and can be distinguished from public services in other fields. Therefore, it is considered that the expression of “sports public service” is more accurate. Aman V. has a different understanding of the concept of sports public service due to different emphases, which can be roughly divided into two types: one is to emphasize the universality of sports service supply mode and the diversity of audiences from the perspective of “publicity” [7]. In order to meet the needs of public sports, the process of providing sports equipment to the public by different governments and institutions is a kind of sports service; secondly, from the perspective of “service,” sports services are government functions. Al A. believes that public sports are a way of meeting the needs of the public and an essential service provided to the public. From the existing research, scientists have different interpretations of public sports due to different viewpoints [8]. The existing research on sports public service is mostly qualitative research, the research results lack certain universality and operability, and the practical guiding significance is not strong. Kim I. g. generally tends to take the government as the leading role in the research on the supply mode, give play to the role of sports intermediary organizations, and make a slow transition to marketization. Macroqualitative research can provide some useful references for the practice of sports public service, but it can not help the deficiency of sports public service system innovation [9]. In addition to macroscopic research, microscopic research also needs to be strengthened. At present, most of the research focuses on the development of sports public services in different regions, cities, and rural areas, and there are few studies on sports public services for multiple groups in the same region, and only a few studies have been heard. Improve the participation of migrant workers and migrants in community public services and sports. Kalman K. believes that people in the same area will have some similarities in their applications for public sports services. Using regions as research data, a broad range of policies to improve physical activity in the public service sector can be obtained. Courses are always carried out at different levels and modes, and in-depth thinking and experience are common and universal so as to provide ideas and applications for improving public physical exams. Therefore, it is necessary to strengthen the research on the size of public sports, which is in line with the reality of urban differences and culture in our country [10].

From a scientific point of view, scientists do more research on government sports programs and less on public needs. Currently, a number of studies have been carried out on the provision of sports services to the public from the perspective of public needs. Asmara, UA paid more attention to the research with the government as the main supplier, ignoring the research and development of public sports applications to public services [11]. Given the important role governments play in providing public sports services, exploring existing resources and providing these types of public sports services from a government perspective can promote the construction and improvement of sports public services to a certain extent. However, the object of sports public service supply is the public. Bekerom, P. said that if the investigation of public demand is not paid attention to, it is easy to lead to the inconsistency between the government's supply and the public's demand, which will lead to the fact that the government has done a lot of work in the supply of sports public services but failed to obtain the public's recognition [12].

The balance of public sports refers to the allocation of sports resources to meet the needs of the public for sports activities. Tan Zhongwei conducted in-depth research on the balance of public sports and believed that the government should play a good role in supervising and creating a good urban and rural environment, city and rural public service activities, and ultimately achieve a balance between urban and rural public service supply and demand [13]. At present, in the research of China's urban and rural public service equation, scientists often choose to study China's urban and rural urban public service equation through theoretical modeling, evaluation modeling, and measurement design. These studies provide a theoretical basis for the equalization of urban and rural sports public services in China. Achieving the balance of sports between urban and rural areas is not only the need to improve social cohesion but also the needs of the rural population for sports. Therefore, it is important to pay attention to the balance of urban and rural public services in the short term. Competitive sports, as a part of the entertainment sports industry and an indispensable part of the sports industry, are gradually recognized and sought after by experienced people. Olympic prowess and athletics have risen rapidly. In some developed countries in Europe and America, the sports industry, especially the competitive sports industry, has become an important part of the national economy. In addition, by analyzing the market performance of the five Olympic Games (23, 24, 25, 26, and 27), some scholars believe that hosting the Olympic Games can create benefits for their country, as shown in Table 1.

## 3. Method

### 3.1. Analysis of Annual Document Volume

The annual distribution of paper output represents the historical context, present, and trend of this research field. As can be seen from Figure 2, the overall research on sports public service in China shows the characteristics of rapid development and fluctuation [14]. The project can be divided into three phases: the “research” phase, the “study” phase, and the “impletement” phase, of which the “research” phase was started from 2007. By 2007, with the improvement of people's daily needs, my country gradually turned the focus of sports science research to the public, and the research began to focus on the analysis of the concept of public sports. The second is the rapid growth stage (2008–2015), the overall rapid growth. The sports public service system in the post-Olympic era has attracted extensive attention. In the period of fluctuating development (from 2016 to now), the literature output decreased significantly in 2016 and did not form a development trend of stable growth, reflecting the lack of sustained research and attention on sports public services in academic circles [15]. In the era of sports power, academia and society should pay attention to this field, as shown in Figure 2.

To understand the backbone of a field, it is generally necessary to explore the core authors in the field and understand them so as to grasp the development status and prospects of the field to a certain extent [16]. According to price's law formula: *N*1 = 0.749 (*N*_max_) 1/2, N1 is the number of papers published at least, *N*_max_ is the scholar with the highest number of papers published, and only the author who reaches N1 can be regarded as the core author. Among them, Wang Jiahong issued 21 articles, that is, *N*_max_ = 21, then *N*1 = 3.4. Therefore, authors with more than 4 articles in this field can be included in the core author group. According to statistics, there are 84 main authors with a total of 580 sentences, accounting for 64% of all publications published by the public service, with more than 50% policy value, indicating that the author is very important. The group was established in the field of Chinese public service sports research [17].

84 *∗* 84 core author co-occurrence matrix is generated through SATI3.2, and the network structure diagram of core author is generated by ucinet6 software. The core author cooperation network is a subnetwork formed by 84 core authors sending documents alone or jointly. In other words, these core authors have great “power” in this field. They hold more resources in this field. They play an important role in resource sharing and information exchange. Generally speaking, it has a certain position or right in this field, which not only depends on the number of documents issued but also plays an important “intermediary” role in scientific research cooperation [18], as shown in Table 2.

Through the statistical software COOC1.7, the documents issued and cooperation of research institutions are statistically analyzed. From Table 3, it can be seen that 48 articles issued by a university occupy the first place, and a university is in the absolute core position in the field of sports public service research. For the cooperation of various institutions, select the institutions with more than 5 documents for visual analysis, finally generate 65 *∗* 65 cooccurrence matrix, and generate the cooperation relationship diagram by using ucinet6 software [19]. It reflects that the overall cooperation relationship is generally close, and a spider web prototype network structure chart with a university as an important node of cooperation has been preliminarily formed, which proves that the cooperation relationship between research institutions in this field is good. Through the statistical analysis of SATI3.2, it is found that 903 papers are distributed in 71 journals, including 40 journals with one article, 19.7% journals with 2–9 papers, and 17 journals with more than 10 papers. The citation frequency of papers is an important index to measure the research ability and paper level of scholars. The higher the citation frequency, the stronger the influence of papers and the higher the academic status and authority of scholars. The cited documents are mainly concentrated in the early 21st century, which is also closely related to the background of building a well-off society in an all-round way and building a socialist harmonious society. During this period, the structure, development, and thinking of the concept of public sports service were examined, which laid the foundation for perfecting thinking in this field. These letters are preceded by 547 letters. The title of this paper is the concept of sports serving the public, which reflects the hotspot of public sports research to a certain extent, as shown in Tables 3 and 4.

### 3.2. Selection of High-Frequency Keywords

Keywords can reveal the research content characteristics, development context, and development trend of a certain field. Use COOC1.7 to extract the keywords, preliminarily process the keywords, delete the keywords that are of little significance to this study, such as “countermeasures,” “current situation,” and “path,” and merge some keywords with similar significance, such as “public sports service” and “public service” into “sports public service,” using the proposed high-frequency keywords, as shown in formula (1). That is, the first 47 keywords are high-frequency keywords, and the frequency of the 48th keyword and the 47th keyword is the same as 8. Therefore, the first 48 keywords are selected as the analysis sample [20], as shown in formula (1) and Table 5.

(1) $$\begin{array}{c} T=47. \end{array}$$

The 48 *∗* 48 cooccurrence matrix formed by 48 high-frequency keywords is processed, the network structure diagram is drawn by using ucinet6 software, and its network density and centrality are analyzed. After calculation, the network density in this field is 0.2646, which is small, indicating that the relationship between keywords is not very close, reflecting less interaction of knowledge content points in this field, and the research content is extensive but not concentrated. Centrality reflects the importance of each keyword in the overall network. If a node is connected with many other nodes, it indicates that this node occupies a central position in the overall network, and the value of centrality is also high [21].

It can be seen from Table 5 that the point degree centrality represents the position of the node in the network structure. The higher the value is, the more likely the keyword will appear. Hot topics such as sports management, public welfare sports, community sports, and major sports are the current research hotspots. Intermediary centrality reflects the influence of keywords on other keywords in the whole network. The greater the value, the greater the bridge function of this keyword. Sports management, community sports, sports public service system, and equalization have high intermediary centrality, which shows that these keywords have a good intermediary role in the network. Proximity centrality reflects the average distance between keywords. The lower the value, the more important the position in the network. Sports management, sports public service system, community sports, etc., have a short distance from other keywords and are close to the center, indicating that these keywords have an important position in the network [22], as shown in Table 6.

Firstly, the 48 *∗* 48 high-frequency keyword cooccurrence matrix is constructed, and then the keyword network structure diagram is drawn by using ucinet6, as shown in Table 7.

Five kinds of word groups are generated through k-core analysis, among which the red word groups are sports public service, community sports, supply, rural, equalization, supply side reform, stadiums and gymnasiums, national fitness, sports management, sports public service system, mass sports, rural sports, sports governance, rural sports public service, resource allocation, sports power, public sports, government functions, competitive sports, and sports industry as the core research hotspot; The second category is marked in blue, focusing on the government, government purchase, sports economy, social sports organizations, service supply, sports associations, policies, and other topics; The third category is marked by black, mainly including Britain, performance evaluation, evaluation index system, Shanghai, system, satisfaction, youth sports, sports sociology, and service-oriented government; The fourth category is pink signs, including government purchase services, urban community sports public services and operation mechanism. The last category is green, which is mainly the concept of sports public service. On the whole, some keywords are at the center of the network, indicating that these topics are the research hotspots in this field, and the keywords at the edge of the network are also the subject areas that scholars need to break through [23].

The number of articles in a journal refers to the number of research documents published in a journal in a certain period of time. By analyzing the distribution of the number of periodicals carrying research literature in a discipline or field, we can determine the core periodicals or core periodical groups of the discipline or field. It is convenient to further understand the spatial distribution of literature in different journals and provide a directional reference for researchers to select journals, publish academic achievements, and grasp research hotspots and research frontiers.

In order to understand the periodical distribution law of academic documents in the field of sports tourism research in China in recent 15 years, the periodical sources of all 464 selected documents were statistically analyzed by using the regional description method and image description method of Bradford's law. Among them, the average article density in the core area and related areas is much higher than the average value, and the discrete area accounts for more than 50% of the total number of journals, but the average article density is far from the average value, which basically conforms to the regional expression of Bradford's law, as shown in Table 8.

The functional relationship between the logarithm of cumulative journals and literature mathematics is shown in Figure 3.

In China, many scientific research achievements are produced in the field of sports sociology every year. Most of these achievements are presented in the form of papers. The distribution relationship between the number of published papers and time has two meanings. On the one hand, it can reflect the development speed and theoretical level of research in this field; On the other hand, according to the annual publication trend of his papers, he can further predict the future development trend and cutting-edge hotspots in this field. The broken line chart of the annual number of documents issued by China's sports sociology is shown in Figure 4.

Through the research, it is found that the realization of network governance of sports public service is different from the traditional single supply mode. Diversified supply subjects, trust, equal communication and coordination mechanism, and long-term repeated game cooperation are its important characteristics. Based on the research, the network model of community sports public service is preliminarily constructed [24], as shown in Figure 5.

The change curve of the number of Sports Tourism Documents in China from 2013 to 2022 is shown in Figure 6.

In the process of internal integration, it should be found that the success of the whole network governance process depends on the cooperation and participation of multiple subjects, and the important variables of their cooperation and participation are the relationship generated and maintained. However, the multisupply subject relationship of sports public service is built on maintenance, which is not only affected by the dimension of relationship quality, but also affected by many other factors. Then, the realization of sports public service supply network governance not only needs the integration of internal resources and the improvement of the relationship quality between subjects but also needs the correct treatment of the factors affecting their interaction [25], as shown in Figure 7.

### 3.3. Lack of Research on Sports Public Services for Special Groups

Special groups refer to groups with special responsibilities. They are vulnerable groups, including the elderly, persons with disabilities, rural marginalized women and children, and marginalized groups. The government should give these groups the right to special attention and attention. Public sports need to ensure that different groups of people get the same level of sports coverage, and the concept of “sports people's lives” needs to be considered in the development of public sports. Due to the limited capacity of the government, the public's interest in participating in the public sports services of professional groups is not strong, and the public services for the pregnancy of professional groups are weak. Now, China's aging and urban economy are getting faster and faster, and the population of elderly, rural backward children, and women is slowly increasing. The protection of special teams' sports rules has not attracted much interest in the educational community [26]. Scholars also lack in-depth investigation and research on the system and mechanism problems encountered by the state in promoting the equalization of sports public services for all groups.

On the premise of establishing a standardized knowledge base and knowledge element, according to the above common situational assumptions, in order to directly operate the knowledge element, it is necessary to transform the technical knowledge demand into a quantifiable star model. Therefore, this paper attempts to propose two groups of new concepts.

The first group of concepts is N(s) and n(s), where n(s) represents the number of knowledge element attribute structures. For a complete knowledge database, the number of structures in which knowledge element information is stored can be quantified and has a fixed value. For example, the columns designed for exclusive data in the database are quantitative, and n(s) represents the number of structures composed of technical problem solutions provided by users according to their own needs and characteristics. Therefore, Ni(s) represents the number of structures of the i-th possible knowledge element in the knowledge set, and ni(s) represents the number of possible knowledge element structures of the problem solution provided by I users in the process of approaching the technical problem demand solution. If the user is more clear about the problem solution structure attribute itself, the number of possible problem solution structures provided will increase. If the number of attributes exceeds the number of knowledge elements, the knowledge element structure may not meet the user's needs or supplement the subclass of demand solutions.

The second group of concepts is N(T) and n(t), where N(T) represents the number of attribute keys contained in the knowledge element content in the knowledge set, n(T) represents the number of attribute keys of the required knowledge content provided by the user, and Ni(T) and ni(t) are similar to those defined in the first group of concepts. Similarly, when the user provides more content keywords about the demand knowledge, the more likely it is to approach the knowledge solution of the demand, but when there are too many content keywords, the mismatch of knowledge elements or the change of dependency relationship of knowledge elements may occur.

Based on the concepts of the number of knowledge element structure items and the number of knowledge element content attributes, combined with the above assumptions, the mathematical model of technical knowledge service is established as follows:

(1) Knowledge element structure containment: in the fuzzy knowledge set, when the structure quantity of *i* knowledge element itself is greater than or equal to a certain proportion of the demand knowledge solution structure quantity of I user demand or submitted by *i* user according to preference, the knowledge structure containment is considered optional, as shown in the following formula:
  (2) $$\begin{array}{c} a\left(i\right)N_{i}\left(S\right)\geq n_{i}\left(s\right). \end{array}$$
a (*i*) is the matching proportion coefficient of knowledge element I corresponding to user I at the knowledge tree structure point, which can be selected appropriately.
(2) Knowledge element content attribute containment. In the fuzzy knowledge set, when the number of possible solution I knowledge element primary key attributes is greater than or equal to a certain proportion of the number of user requirements or the number of demand knowledge solution content primary key attributes submitted by I users according to their preferences, it is considered that knowledge matching is optional, as shown in the following formula:
  (3) $$\begin{array}{c} b\left(i\right)N_{i}\left(T\right)\geq n_{i}\left(t\right). \end{array}$$
b(*i*) is the matching proportion coefficient of knowledge element I corresponding to user I in the primary key of the knowledge tree content attribute, which can be selected appropriately.
(3) Knowledge is available. When the structure and content of knowledge are based on the above conditions, and the result at least meets the user's expectations for the knowledge structure and content of problem solving, knowledge content is the goal of success. At the same time, in order to control falling into local fraud scenarios, the solution is further limited to include various problem solving techniques, when it comes to higher than standard requirements, as shown in the following formulas:
  (4) $$\begin{array}{c} \text{Max}\left[a\left(i\right)N_{i}\left(S\right)-n_{i}\left(s\right)\right]+\left[b\left(i\right)N_{i}\left(T\right)-n_{i}\left(t\right)\right]. \end{array}$$
  (5) $$\begin{array}{c} \sum_{i=1}^{n}\left[a\left(i\right)N_{i}\left(S\right)+b\left(i\right)N_{i}\left(T\right)\right]\geq \sum_{i=1}^{n}\left[n_{i}\left(s\right)+n_{i}\left(t\right)\right]. \end{array}$$
  (6) $$\begin{array}{c} a\left(i\right)N_{\text{max}}\left(S\right)\geq a\left(i\right)N_{i}\left(S\right). \end{array}$$
  (7) $$\begin{array}{c} a\left(i\right)N_{i}\left(S\right)\geq n_{i}\left(s\right). \end{array}$$
  (8) $$\begin{array}{c} b\left(i\right)N_{\text{max}}\left(T\right)\geq b\left(i\right)N_{i}\left(T\right). \end{array}$$
  (9) $$\begin{array}{c} b\left(i\right)N_{i}\left(T\right)\geq n_{i}\left(t\right). \end{array}$$
  (10) $$\begin{array}{c} N_{i}\left(S\right)=\sum_{i=1}^{\text{it}}N_{ij}\left(S\right). \end{array}$$
  (11) $$\begin{array}{c} N_{i}\left(T\right)=\sum_{i=1}^{\text{it}}N_{ij}\left(T\right). \end{array}$$

For formula (4), if the objective function is to find the optimal solution, the problem solution will become the only solution, which obviously loses the initiating characteristics of the knowledge solution. Therefore, in order to maintain the heuristic of the solution, the selected knowledge elements with better isomorphism and better content matching should be collected to generate knowledge blocks of the appropriate size to prepare for the operation of knowledge fusion gene fragments. Find the optimal value of the gene block containing the number of knowledge elements C (the smaller its accuracy is, the higher the heuristic knowledge solution may be, and it will lose significance in macro). Therefore, in order to obtain the optimal knowledge block, the objective function is obtained after deformation, as shown in the following formulas:

(12) $$\begin{array}{c} \text{Min}\left[cn_{i}\left(s\right)-\sum_{i=1}^{n}a\left(i\right)N_{i}\left(S_{j}\right)\right]+\left[cn_{t}\left(t\right)-\sum_{i=1}^{n}b\left(i\right)N_{i}\left(T_{j}\right)\right]. \end{array}$$

(13) $$\begin{array}{c} \sum_{i=1}^{n}\left[a\left(i\right)N_{i}\left(S\right)+b\left(i\right)N_{i}\left(T\right)\right]\geq \sum_{i=1}^{n}\left[n_{i}\left(s\right)-n_{i}\left(t\right)\right]. \end{array}$$

(14) $$\begin{array}{c} a\left(i\right)N_{\text{max}}\left(S\right)\geq a\left(i\right)N_{i}\left(S\right)\geq n_{i}\left(t\right). \end{array}$$

(15) $$\begin{array}{c} b\left(i\right)N_{\text{max}}\left(T\right)\geq b\left(i\right)N_{i}\left(T\right)\geq n_{i}\left(s\right). \end{array}$$

(16) $$\begin{array}{c} N_{i}\left(S\right)=\sum_{i=1}^{\text{it}}N_{ij}\left(T\right). \end{array}$$

(17) $$\begin{array}{c} N_{i}\left(T\right)=\sum_{i=1}^{it}N_{ij}\left(S\right). \end{array}$$

## 4. Results and Analysis

With the gradual advancement of rural development and rural revitalization strategies, the research on rural sports by professionals and scholars has gradually increased. In recent years, although my country's public sports services have achieved success, there is still a big difference between the quality and quantity of rural public sports in my country and the needs of the rural masses [27]. China's rural sports public service scientific research is also emerging. The researchers conducted in-depth research on the significance, existing problems, and protection of rural sports in our country. Research shows that the rural sports public service in my country has a negative impact on the development of sports facilities, the number of sports coaches, managers, and the number of people engaged in sports activities. The government should increase its support for the development of rural sports.

Under the background of rural revitalization, my country's rural structure has undergone major changes, gradually changing the main body from individual farmers to a new situation in which many factors, such as immigrants and farmers, work together. The change of rural mass identity makes the supply object of rural sports public service become complex. Different objects have different sports needs. Scholars should pay attention to how to adjust the supply mode to meet the sports needs of different objects [28]. In addition, under the social background of sports power, how to strengthen the supply of rural sports facilities, how to improve the supply structure of rural sports public service, and how to serve different supply objects will also be the focus of the research on the supply of rural sports public service in the future.

Based on the background of the information age, the integration of information networks and the development of public services have created opportunities to support the modernization of informatization and public sports. Smart sports services should reflect current characteristics, meet public sports needs in principle, affect sports equipment and sports expertise, and be used for public works, monitoring, and evaluation. The research and development of sports to public services such as the Internet, cloud computing, 5G technology, and other information networks requires comprehensive research, and cooperative research in this field will continue in the future.

The central and local governments have unclear rights and responsibilities and overlapping functions in the field of sports public services. The responsibilities and rights of some sports public services do not match the financial capacity of local governments. At this stage, to strengthen the construction of sports public service, we must accurately define the sports public service functions of the central government and local governments. Not all sports public services need the intervention of governments at all levels. Therefore, the research on sports public service must clarify the responsibilities of sports public service between governments at all levels and strengthen the research on the responsibilities of sports public service between governments at all levels.

The public sports model is an important basis for the balance of urban and rural sports. To measure the effectiveness of public sports services, we need to develop appropriate, researched models of public sports services. The development and implementation of public sports service models can support the development of high-quality public health services. The landscape of public service sports has not changed. Local government departments should clarify the minimum standards of sports public services such as sports facilities services and sports activities services according to the economic and social development of the region and implement them widely in the region. Therefore, from the perspective of understanding the differences between urban and rural areas, East and West, combined with the current situation of public services in multiple regions, through research and demonstration, the public sports service model will be developed. After the design, through continuous efforts, the gap between urban and rural areas and the eastern and western regions in public sports will be gradually narrowed so that most people can realize the importance of public sports and complete public services, to achieve the goal of equalization of sports public services as soon as possible.

Performance evaluation of sports public services, as an effective entry point for government management decision-making and function transformation, has attracted widespread attention from local governments at all levels and academics. In the field of research on sports public services in China, most scholars have conducted more research on supply subjects, supply content, and people's needs, while less research has been conducted on the performance evaluation of sports public services. Research on the evaluation of the performance of sports public services in China can raise the government's awareness of the importance of sports public service supply and institutional construction. By studying the content, evaluation index system, and evaluation methods of sports public service performance evaluation, a wide range of scholars can promote the systematization and standardization of sports public service management and further promote the transformation of government functions.

## 5. Conclusion

It proves that the problem of promoting public sports service research based on measurement data in my country can be solved. Give play to the role of public services and improve the people's enjoyment of public services. There are big differences in the development of public service sports in my country. Uncertainty in development often occurs in eastern and western regions, between urban and rural areas, and between groups. Equitable access to public sports services has always been a goal set by governments at all levels. At present, China is still exploring ways and means to achieve a balance in public sports services. The majority of scholars should strengthen the research on the equalization of sports public services for vulnerable groups, urban-rural fringe, and rural poor areas, and timely summarize the experience in the process of realizing the equalization of sports public services outside China, which has important theoretical and practical significance for China to achieve the goal of equalization of sports public services as soon as possible.

## Figures and Tables

**Figure 1:** Development process of Chinese sports.

**Figure 2:** Annual distribution of literature in the field of sports public service research.

**Figure 3:** Functional relationship between logarithm of cumulative journal quantity and literature mathematics.

**Figure 4:** Quantity trend of sports sociology research literature in China from 2013 to 2022.

**Figure 5:** Community sports public service network model.

**Figure 6:** Number and year distribution of sports tourism research literature in China from 2013 to 2022.

**Figure 7:** Elements of network governance.

**Table 1:** Economic benefit ratio of the 23rd–27th Olympic Games (unit: USD 100 million).

Session	Time	Economic benefit ratio
23	1984	1.55
24	1988	1.60
25	1992	1.00
26	1996	1.00
27	2000	1.83

**Table 2:** Number of articles published by core authors (top 15).

Number of documents issued	Number of documents issued	Number of documents issued
21	13	11
21	13	11
15	12	11
15	11	11
11	11	11

**Table 3:** Distribution of periodicals.

Periodical	Number of publications
Sports culture guide	107
Journal of physical education	51
Sports and science	49
Journal of a sports college	55

**Table 4:** Highly cited literature in the field of sports public service research.

Paper	Particular year
Concept and theoretical analysis of public sports service	2020
Discussion on the concept development and structure of China's public sports service system	2019
Building a perfect sports public service system	2020
Application and analysis of PPP mode in the field of public services	2018

**Table 5:** High-frequency keywords.

Key word	Frequency/time
Sports public service	677
Sports management	88
Sports public service system	60
Equalization	55
Government purchase	53
Mass sports	48
Stadium	45
Social sports organization	42
Community sport	42
National fitness	41
Supply	39
Rural sports	33
Government	30
Satisfaction	23
Rural sports public service	20
Governmental functions	19
Supply side reform	19
Countryside	19
Public sports	18
Sports economy	18
Evaluation index system	18
Sports governance	16
Service supply	14
Resource allocation	14
System	13
Sports power	12
Sports sociology	12
Healthy	12
Policy	12
Pattern	12
Demand	11
Government purchase of services	11
Sport industry	10
Sports rights	10
Britain	10
Competitive sports	10
Supply subject	10
Service-oriented government	9
Youth sports	9
Operating mechanism	9
Reform	9
Urban community sports public service	8
Disabled	8
Social sports	8
Sports associations	8
Performance evaluation	8
Concept	8
Structure	8

**Table 6:** Centrality analysis of high-frequency keywords (part).

Serial number	Keyword	Point degree centrality	Intermediary centrality	Near centrality
1	Sports public service	46	321.45	46
2	Sports management	31	75.46	61
3	Sports public service system	24	49.22	68
4	Community sport	23	51.01	69
5	Mass sports	22	26.47	70
6	National fitness	19	21.66	73
7	Stadium	18	23.69	74
8	Equalization	18	26.21	74
9	Government purchase	16	20.21	76
10	Rural sports	16	12.97	76
11	Supply	16	19.67	76
12	Public sports	15	13.23	77
13	Governmental functions	15	7.46	77
14	Sports governance	15	9.27	77
15	Social sports organization	14	13.88	78

**Table 7:** High-frequency keyword cooccurrence matrix (part).

Key word	Sports public service	Sports management	Sports public service system	Equalization	Government purchase
Sports public service	0	69	9	41	51
Sports management		0	5	4	7
Sports public service system			0	0	0
Equalization				0	0
Government purchase					0

**Table 8:** Regional statistics of core journals in China's sports tourism field from 2000 to 2014.

Partition	Number of periodicals	Number of documents (articles)	Zai Wenbi (%)	Proportion in the total number of journals (%)	Average document density (articles/kind)
First area (core area)	3	171	36.85	17.65	57
Second area (relevant area)	5	163	35.13	29.41	33
Third area (discrete area)	9	130	28.02	52.94	14
Total	17	464	100	100	27

## Data Availability

The labeled data set used to support the findings of this study is available from the corresponding author upon request.
